The article "Secure Complex Systems: A Dynamic Model in the Synchronization" was retracted in 2023. Reasons: signs of a paper mill; suspected computer-generated content; unreliable results or conclusions; concerns about the data.

# Secure Complex Systems: A Dynamic Model in the Synchronization

**DOI:** 10.1155/2021/9719413

**Published:** 2021-12-23

**Authors:** Abdulsattar Abdullah Hamad, M. Lellis Thivagar, Jalawi Alshudukhi, Talal Saad Alharbi, Saud Aljaloud, Khalid Twarish Alhamazani, Zelalem Meraf

**Affiliations:** ^1^College of Sciences, Tikrit University, Tikrit, Iraq; ^2^School of Mathematics, Madurai Kamaraj University, Madurai, Tamilnadu, India; ^3^University of Ha'il, College of Computer Science and Engineering Department of Computer Science, Ha'il, Saudi Arabia; ^4^Department of Statistics, Injibara University, Injibara, Ethiopia

## Abstract

Chaotic systems are one of the most significant systems of the technological period because their qualities must be updated on a regular basis in order for the speed of security and information transfer to rise, as well as the system's stability. The purpose of this research is to look at the special features of the nine-dimensional, difficult, and highly nonlinear hyperchaotic model, with a particular focus on synchronization. Furthermore, several criteria for such models have been examined; Hamiltonian, synchronizing, Lyapunov expansions, and stability are some of the terms used. The geometrical requirements, which play an important part in the analysis of dynamic systems, are also included in this research due to their importance. The synchronization and control of complicated networks' most nonlinear control is important to use and is based on two major techniques. The linearization approach and the Lyapunov stability theory are the foundation for attaining system synchronization in these two ways.

## 1. Introduction

The Lyapunov method, which is referred to as the Lyapunov stability criterion, uses a Lyapunov *V*(*x*) function that is similar to the potential function of classical dynamics. It is given as follows for a system (*x*  = *f*(*x*)) that has an equilibrium point at *x* = 0. In the recent past, the study of nonlinear continuous dynamical systems has been considerable. It is one of the first trials in the Lu model [1]. It presents the new structure of high dimension (9D), novel king of quaternion complete, and has some unusual properties [2–4]. There is another study, which introduces another chaotic and hyperchaotic complex nonlinear, and this type has and its phase-space behavior holds a great amount of weight [6–9]. It was previously structured, for example, a three-dimensional auto system that is not differ-isomorphic with the Lorenz attractor. Lü [10] presented another 3D attractor that is chaotic in different ways and is not diffeomorphic with Lorenz [3, 4, 11, 12] in terms of the arrangement of values for a parameter *k*. Lorenz [5], an extension of the Lorenz system, proposed the first chaotic nonlinear system. The mechanics of liquid flows' calorific convection are simulated using the Lorenz system's messy structure [13]. Many chaotic and super-chaotic complex systems with nonlinear quadratic conditions have been proposed in [13–15]. The Lorenz equation is used to combine these systems with nonlinear quadratic components. In the suggested model, the variables *x* and *y* are taken to be functions for one real and three complex parameters. It was previously structured; for example, a three-dimensional auto system that is not differ-isomorphic with the Lorenz attractor. Lü has suggested another 3D attractor that exhibits chaotic behavior in different ways and is not diffeomorphic with Lorenz in terms of the arrangement of values for a parameter *k*.

The article "Secure Complex Systems: A Dynamic Model in the Synchronization" was retracted in 2023. Reasons: signs of a paper mill; suspected computer-generated content; unreliable results or conclusions; concerns about the data.

The *z* variable, on the contrary, can only be predicted using real variables. A set of nine equations illustrates the hypercomplex chaotic system after extensive mathematical modifications. The collected system dynamics were examined, including phase spaces, eigenvalue computations, and Lyapunov exponent calculations, as well as all other studies. When compared to the findings obtained with 6D models, the suggested approach reveals an acceptable level of accuracy. Several research publications have attempted to look into the geometry of nature, complex-dynamic network synchronization, and regulation of specific topologies. It can be assumed that the three-following 1st O.D.E. characterizes a model proposed by Alyami and Mahmoud [5]. Lots of systems have been studied such as 2D, 3D, 4D, and 8D.

In this paper, we will present a study on a proposed model 9D and try to verify its validity, as the mathematical equations will be mentioned in sequence.

### 1.1. Contribution

- We have proposed the system which clearly depicts that while increasing the parameter, the corresponding values of are decreased
- From a detailed analysis and results, we have achieved featured for the 9-dimensional, complex, and highly nonlinear hyperchaotic model which has been executed to make a model more dynamic
- For various models, several criteria have been examined, such as Hamiltonian, Synchrony, Lyapunov expansion, and stability

## 2. Structure

In the present section, a short review of the model developed by Lellis, and Hamad is presented to ensure continuity of the concept of the present study.

The system depends entirely on the mathematical equations that enable us to reach numerical results, as the nine-year system is considered one of the most recent and most complex systems. Circuit simulation is a process in which a model of an electronic circuit is created and analyzed using various software algorithms, which predict and verify the behavior and performance of the circuit. Here, we can explain and give the mathematical equations that the system adopts to prove its testability of its validity:

(1) $$\begin{array}{c} \overset{•}{x\left(t\right)}=\alpha \left(y-x\right), \end{array}$$

(2) $$\begin{array}{c} \;y^{.}\left(t\right)=\left(\gamma x-y-xz\right), \end{array}$$

(3) $$\begin{array}{c} \overset{•}{z\left(t\right)}=-\beta z+\frac{1}{2}\left(y\bar{x}+x\bar{y}\right), \end{array}$$

where *α*, *β*,  and *γ* are real parameters, and the variables *x*, *y*,  and *z* are defined as

(4) $$\begin{array}{c} x=u_{1}+iu_{2}+ju_{3}+ku_{4}, \end{array}$$

(5) $$\begin{array}{c} y=u_{5}+iu_{6}+ju_{7}+ku_{8}, \end{array}$$

(6) $$\begin{array}{c} z=u_{9}. \end{array}$$

The complex variables were calculated using the traditional Lu Model. It may be deduced from the given model that the model was created by replacing actual variables. This is seen in equations (4) and (5). The system has been proposed and achieved at large sizes. Two alternative strategies are intended to be used to build a higher-dimensional model, which may be accomplished by adding additional variables to the first system's original system. It takes into account the second by integrating two existing models in order to produce a stable system. This procedure requires extra caution. It is the initial way that has been picked to create the present process in this text.

The article "Secure Complex Systems: A Dynamic Model in the Synchronization" was retracted in 2023. Reasons: signs of a paper mill; suspected computer-generated content; unreliable results or conclusions; concerns about the data.

Equations (1) through (2) are treated mathematically; equations (4) and (5) are substituted into both sides of equation (1) as follows:

(7) $$\begin{array}{c} {\overset{•}{u}}_{1}+i{\overset{•}{u}}_{2}+j{\overset{•}{u}}_{3}+k{\overset{•}{u}}_{4}=\alpha \left(\left(u_{5}+iu_{6}+ju_{7}+ku_{8}\right)-\left(u_{1}+iu_{2}+ju_{3}+ku_{4}\right)\right). \end{array}$$

Both sides have been the manipulation of equation (7), and after a long mathematical, the first-order differential equation will get it from the following system:

(8) $$\begin{array}{c} {\overset{•}{u}}_{1}=\alpha \left(u_{5}-u_{1}\right),\\ {\overset{•}{u}}_{3}=\alpha \left(u_{7}-u_{3}\right),\\ {\overset{•}{u}}_{4}=\alpha \left(u_{8}-u_{4}\right),\\ {\overset{•}{u}}_{5}=\gamma u_{1}-u_{5}-u_{1}u_{9},\\ {\overset{•}{u}}_{6}=\gamma u_{2}-u_{6}-u_{2}u_{9},\\ {\overset{•}{u}}_{7}=\gamma u_{3}-u_{7}-u_{3}u_{9},\\ {\overset{•}{u}}_{8}=\gamma u_{4}-u_{8}-u_{4}u_{9}, \end{array}$$

(9) $$\begin{array}{c} {\overset{•}{u}}_{9}=-\beta u_{9}+\left(u_{1}u_{5}+u_{2}u_{6}+u_{3}u_{7}+u_{4}u_{8}\right). \end{array}$$

### 2.1. Hamiltonian Dynamics

In this section, in particular, the study considers the system smooth and nonlinear; then, it is generalized, and the Hamiltonian canonical form takes the following way:

(10) $$\begin{array}{c} \overset{•}{\chi }\left(x\right)=\tau \left(x\right)\frac{\partial H}{\partial x}+S\left(x\right)\frac{\partial H}{\partial x},\;x\in R^{n}. \end{array}$$

In equation (9), *H* is a smooth energy function.

The article "Secure Complex Systems: A Dynamic Model in the Synchronization" was retracted in 2023. Reasons: signs of a paper mill; suspected computer-generated content; unreliable results or conclusions; concerns about the data.

The vector-matrix on the right-hand side is the primary system itself; therefore, the Hamiltonian takes the following form:

(11) $$\begin{array}{c} \overset{•}{\chi }\left(x\right)=\frac{1}{2\alpha }\left[U_{1}^{2}+U_{2}^{2}+U_{3}^{2}+U_{4}^{2}+U_{5}^{2}+U_{6}^{2}+U_{7}^{2}+U_{8}^{2}+U_{9}^{2}\right]. \end{array}$$

Equation (10) is the new Hamiltonian.

### 2.2. Symmetry and Invariance

Both are invariant because of the invariance:

(12) $$\begin{array}{c} u_{1},u_{2},u_{3},u_{4},u_{5},u_{6},u_{7},u_{8},u_{9}, \end{array}$$

(13) $$\begin{array}{c} -u_{1},-u_{2},-u_{3},-u_{4},-u_{5},-u_{6},-u_{7},-u_{8},-u_{9}. \end{array}$$

It can be proven that there are two solutions by the following substitution by introducing

(14) $$\begin{array}{c} \left\{\begin{array}{c} u_{K}^{/r}=u_{K}^{/r}\cos\;\Theta -u_{K}^{/i}\sin\;\Theta ,\\ u_{K}^{/i}=u_{K}^{/i}\sin\;\Theta +u_{K}^{/i}\cos\;\Theta ,\;k=1,2,3,\ldots ,9. \end{array}\right. \end{array}$$

 
*r*: real
 
*i*: imaginary
 
*k* = 1, 2, 3,…, 9

### 2.3. Equilibria

In this section, equilibrium is needed to find the homogenous solution given by the new system by equation (8) as follows:

(15) $$\begin{array}{c} \alpha \left(u_{5}-u_{1}\right)=0\;⟹\;u_{1}=u_{5},\\ \alpha \left(u_{6}-u_{2}\right)=0\;⟹\;u_{2}=u_{6},\\ \alpha \left(u_{7}-u_{3}\right)=0\;⟹\;u_{3}=u_{7},\\ \alpha \left(u_{8}-u_{4}\right)=0\;⟹\;u_{4}=u_{8},\\ \gamma u_{1}-u_{5}-u_{1}u_{9}=0\;⟹\;u_{1}\left(\gamma -u_{9}-1\right)=0,\\ \gamma u_{2}-u_{6}-u_{2}u_{9}=0\;⟹\;u_{2}\left(\gamma -u_{9}-1\right)=0,\\ \gamma u_{3}-u_{7}-u_{3}u_{9}=0\;⟹\;u_{3}\left(\gamma -u_{9}-1\right)=0,\\ \gamma u_{4}-u_{8}-u_{4}u_{9}=0\;⟹\;u_{4}\left(\gamma -u_{9}-1\right)=0,\\ -\beta u_{9}+\left(u_{1}^{2}+u_{2}^{2}+u_{3}^{2}+u_{4}^{2}\right)=0. \end{array}$$

From the 5th row in equation (14) till the 8th row, one can obtain the only possible solution *u*_9_=*γ* − 1; while all remaining variables equal zero, i.e., *u*_1_=*u*_2_=*u*_3_=*u*_4_=*u*_5_=*u*_6_=*u*_7_=*u*_8_=0.

### 2.4. Stability

The authors have referred back to Jacobin, and the study has proposed a system by equation (14) to find characteristic eques as follows to check the stability:

(16) $$\begin{array}{c} \left\|J-\lambda \right\|=\left(\begin{array}{ccccccccc} -\alpha -\lambda & 0 & 0 & \alpha & 0 & 0 & 0 & 0 & 0\\ 0 & -\alpha -\lambda & 0 & 0 & 0 & \alpha & 0 & 0 & 0\\ 0 & 0 & -\alpha -\lambda & 0 & 0 & 0 & \alpha & \alpha & 0\\ 0 & 0 & 0 & -\alpha -\lambda & 0 & 0 & 0 & 0 & 0\\ \gamma & 0 & 0 & 0 & -1-\lambda & 0 & 0 & 0 & 0\\ 0 & \gamma & 0 & 0 & 0 & -1-\lambda & 0 & 0 & 0\\ 0 & 0 & \gamma & 0 & 0 & 0 & -1-\lambda & 0 & 0\\ 0 & 0 & 0 & \gamma & 0 & 0 & 0 & -1-\lambda & 0\\ 0 & 0 & 0 & 0 & 0 & 0 & 0 & 0 & -\beta -\lambda \end{array}\right)=0. \end{array}$$

The article "Secure Complex Systems: A Dynamic Model in the Synchronization" was retracted in 2023. Reasons: signs of a paper mill; suspected computer-generated content; unreliable results or conclusions; concerns about the data.

### 2.5. Dissipation

From the divergence condition and the dissipation of the system, it will be examined follows:

(17) $$\begin{array}{c} \nabla \;•\;V=\sum_{i=1}^{N=9}\frac{\partial {\overset{•}{u}}_{i}}{\partial u_{i}}<0. \end{array}$$

By computing after simplifying partial derivatives, the dissipation condition is as follows:

(18) $$\begin{array}{c} \nabla \;•\;V=-4\alpha -\beta -3=-\left(4\alpha +\beta +3\right). \end{array}$$

It is possible to state that a circumstance is at the root of the occurrence of chaotic behavior.

### 2.6. Lyapunov Exponents

Referring back to the system derived by equation (8) and recasting, it is in a general matrix form, and it will take the following form:

(19) $$\begin{array}{c} \overset{•}{U}\left(t\right)=\xi \left(U\left(t\right);\zeta \right), \end{array}$$

where

(20) $$\begin{array}{c} \zeta ={\left(\zeta_{1},\zeta_{2},\zeta_{3},\ldots ,\zeta_{9}\right)}^{T}. \end{array}$$

Now, it defines the deviation in solving as follows:

(21) $$\begin{array}{c} \delta \overset{•}{U}\left(t\right)=L_{ij}\left(U\left(t\right);\zeta \right)\delta U\left(t\right), \end{array}$$

(22) $$\begin{array}{c} L_{ij}\left(U\left(t\right);\zeta \right)=\frac{\partial U\;{\left(t\right)}_{i}}{\partial u_{j}}, \end{array}$$

(23) $$\begin{array}{c} J_{ij}=\left(\begin{array}{ccccccccc} -\alpha & 0 & 0 & 0 & \alpha & 0 & 0 & 0 & 0\\ 0 & -\alpha & 0 & 0 & 0 & \alpha & 0 & 0 & 0\\ 0 & 0 & -\alpha & 0 & 0 & 0 & \alpha & 0 & 0\\ 0 & 0 & 0 & -\alpha & 0 & 0 & 0 & \alpha & 0\\ \gamma & 0 & 0 & 0 & -1 & 0 & 0 & 0 & 0\\ 0 & \gamma & 0 & 0 & 0 & -1 & 0 & 0 & 0\\ 0 & 0 & \gamma & 0 & 0 & 0 & -1 & 0 & 0\\ 0 & 0 & 0 & \gamma & 0 & 0 & 0 & -1 & 0\\ 0 & 0 & 0 & \gamma & 0 & 0 & 0 & 0 & -\beta \end{array}\right), \end{array}$$

(24) $$\begin{array}{c} \left\|J_{ij}\right\|=\alpha^{4}\beta \left(-\gamma^{4}+4\gamma^{3}-6\gamma^{2}+4\gamma -6\right). \end{array}$$

The choice of the parameters *α*, *β*,  and *γ* determines the hyperchaotic system, and it is essential to remain as it is by increasing the number of positive Lyapunov exponents and the occurrence of the hyperchaotic.

### 2.7. Lyapunov Attractors

As reported by Yorke–Kaplan, the Lyapunov dimension of the dynamic system's attractors is

(25) $$\begin{array}{c} D=\alpha^{*}+\frac{\sum_{K=1}^{\alpha^{*}}L_{ij}}{\left|L_{\alpha^{*}+1}\right|}. \end{array}$$

In equation (24), *α*^*∗*^ is the highest integer for which ∑_*K*=1_^*α*^*∗*^^*L*_*ij*_ should be negative.

The article "Secure Complex Systems: A Dynamic Model in the Synchronization" was retracted in 2023. Reasons: signs of a paper mill; suspected computer-generated content; unreliable results or conclusions; concerns about the data.

### 2.8. Model of a Weighted-Complex Network

In this study, the authors will apply a weighted-complex-dynamic model provided by [6, 9], to the dynamic model they built. The following is what the model suggested:

(26) $$\begin{array}{c} \left\{\begin{array}{c} \frac{\partial y_{j}}{\partial t}=g\left(y_{j}\right)+\sum_{j=1}^{M}C_{ij}\Delta y_{j},\;1\leq i\leq M,\\ y_{j}={\left(y_{i1},y_{i2},y_{i3},\ldots ,y_{im}\right)}^{T}\in R^{n}. \end{array}\right. \end{array}$$

## 3. The Method of Adaptive Control

The identity in this section is regulated by the following:

(27) ∂y^j∂t=gy^j+∑j=1MC^ijΔy^j+ζi, 1≤i≤M,y^j=y^i1,y^i2,y^i3,…,y^imT∈Rn.

By making use of the following assumption,

(28) y¯•=y^j−yj,C¯=C^j−Cj,

the error system formula will take the following form:

(29) y¯•=gy^j−gyj+∑j=1MC¯ijΔyj+∑j=1MCijy¯g+ζi,y¯=y^j−yj,C¯=C^j−Cj.

## 4. Numerical Results and Discussion

In this work, four sets of the parameters *α*, *β*,  and *γ* are tested, and the corresponding Lyapunov exponents are computed. These sets are shown in Table 1, and Table 2 shows numerical values.

Initial conditions:

(30) $$\begin{array}{c} u_{1}\left(0\right)=0.999,\\ u_{2}\left(0\right)=1.999,\\ u_{3}\left(0\right)=2.999,\\ u_{4}\left(0\right)=3.999,\\ u_{5}\left(0\right)=4.999,\\ u_{6}\left(0\right)=5.999,\\ u_{7}\left(0\right)=6.999,\\ u_{8}\left(0\right)=7.999,\\ u_{9}\left(0\right)=8.999. \end{array}$$

By MATLAB software, we will include and analyze the numerical values.

### 4.1. Attractors of a Proposed System

Figures 1 and 2 show studies of the control and synchronization behavior of a particular model are of practical interest. In light of this, the current work focuses on

- Design an adaptive control strategy for the synchronization phenomena of the chaotic system with known and unknown parameters
- Design a nonlinear control function capable of controlling the hyperturbulent system to stabilize any situation and follow any path while being smooth functionality
- Design a control function capable of synchronizing two identical or different chaotic systems evolving under different conditions

## 5. Conclusions

In the present research work, the authors have proposed the system by four different sets for the parameters as shown Tables 1 and 2. The results, due to these sets, are shown in Figures 1-2. As it is clear that while increasing the parameter, the corresponding values decreased on 9D. Dynamic systems are one of the important systems of the era of technology, as the properties of these systems always need to be updated, for the speed of security and information transfer increases as well as the stability of the system. The present study aims to analyze the detailed features of the nine-dimensional, complex, and highly nonlinear hyperchaotic model. Furthermore, various criteria, such as Hamiltonian, synchronization, Lyapunov expansion, and stability, have been investigated for such models.

The article "Secure Complex Systems: A Dynamic Model in the Synchronization" was retracted in 2023. Reasons: signs of a paper mill; suspected computer-generated content; unreliable results or conclusions; concerns about the data.

## Figures and Tables

**Figure 1:** Attractor of the system in the (*u*1, *u*2, *u*3) space.

**Figure 2:** Attractor of the system in the (*u*2, *u*6, *u*9) space.

**Table 1:** Lyapunov exponents.

Parameters (set)	Set (1)	Set (2)	Set (3)	Set (4)
*α*	10	12	14	16
*β*	3.7	4.7	5.7	6.7
*γ*	55	56	57	58

**Table 2:** Numerical values.

	Set (1)	Set (2)	Set (3)	Set (4)
*L*_1_	1.01	1.009	1.005	1.002500
*L*_2_	0.741	0.74050	0.74020	0.740050
*L*_3_	0.41	0.40050	0.40025	0.4000100
*L*_4_	0.141	0.14050	0.14004	0.140025
*L*_5_	0	0.00000	0.00000	0.000000
*L*_6_	−17.0051	−17.0071	−17.0081	−17.0095
*L*_7_	−23.9108	−23.9118	−23.9127	−23.9132
*L*_8_	−70.2753	−70.2761	−70.2753	−70.2772
*L*_9_	−70.3127	−70.3138	−70.3142	−70.3145

## Data Availability

The data used to support the findings of this study are included within the article.
